The article "Effect of Different Breast Densities and Average Glandular Dose on Contrast to Noise Ratios in Full-Field Digital Mammography: Simulation and Phantom Study" was published in 2018. Journal: Radiol Res Pract.

# Effect of Different Breast Densities and Average Glandular Dose on Contrast to Noise Ratios in Full-Field Digital Mammography: Simulation and Phantom Study

**DOI:** 10.1155/2018/6192594

**Published:** 2018-12-10

**Authors:** Noriko Nakamura, Yuka Okafuji, Saori Adachi, Kana Takahashi, Takashi Nakakuma, Sohichirou Ueno

**Affiliations:** ^1^Department of Radiology, Ageo Central General Hospital, Ageo-City, Saitama 362-8588, Japan; ^2^Graduate School of Health Science, Suzuka University of Medical Science, Mie 510-0293, Japan; ^3^Department of Breast Surgery, Ageo Central General Hospital, Ageo-City, Saitama 362-8588, Japan

## Abstract

We aimed to investigate the effects of mammary gland density and average glandular dose (AGD) on contrast-to-noise ratio (CNR) of breast-equivalent phantoms with different mammary gland/fat tissue ratios. Full-field digital-mammography breast X-rays were performed on breast-equivalent phantoms with three different mammary gland/fat tissue ratios (Phantom A [30/70], Phantom B [50/50], and Phantom C [70/30]) and seven thicknesses ranging from 10 mm to 70 mm. The prediction formula for the CNR was calculated by multivariate analysis and the effects of the various parameters on CNR were evaluated using a multiple regression analysis model. Higher CNR values were obtained with lower mammary gland/fat tissue ratios and lower phantom thicknesses. Variation in CNR among the three breast models was low (coefficient of variation, 3.4–8.7%) at lower phantom thicknesses (10–30 mm) and high (coefficient of variation, 10.5–16.8%) at higher phantom thickness (50–70 mm). CNR showed a strong negative correlation (r = -0.8989) with AGD across all three mammary gland ratios. A predictive formula for CNR using AGD and mammary gland density was developed. CNR can be predicted with high precision using AGD and mammary gland density. The predicted CNR could be used to measure the diagnostic reliability of mammography in breast cancer.

## 1. Introduction

Early detection of breast cancer though mammographic screening has significantly reduced breast cancer mortality [1]. Since mammary glands are less permeable to X-rays than fat tissue in the breast, mammography (MMG) essentially creates a contrast image of the breast based on differences in X-ray attenuation by different tissue components [2]. The area ratio of mammary gland tissue to the fat tissue within the entire breast mammogram is referred to as the mammary gland density in MMG. Breast density is a significant factor in the reliability of breast cancer diagnosis for two reasons. Dense breast tissue has not only been demonstrated to be a risk factor for breast cancer in Western [3–9] and Japanese women [10–12], it is also known to reduce the detection sensitivity of breast cancer in clinical settings [13]. Kolb et al. [13] reported that the detection sensitivity of cancer in low-density mammary gland tissue is 83%–98% compared to 48%–64% in dense breast tissue.

The article "Effect of Different Breast Densities and Average Glandular Dose on Contrast to Noise Ratios in Full-Field Digital Mammography: Simulation and Phantom Study" was published in 2018. Journal: Radiol Res Pract.

Considering the importance of breast density in cancer diagnosis and risk evaluation, the American College of Radiology has proposed a Breast Imaging Reporting and Data System (BI-RADS) classification system for standardized interpretation and reporting of mammograms [14]. As per the latest version, lesions are classified into six grades, including two high-risk grades that pertain to highly dense mammary gland breast tissue. Appropriate diagnosis depends not only on proper interpretation but also on good mammogram image quality [15]. Identifying breast cancer in dense breast tissue is challenging because of the masking effect of the mammary glands, which results in poor image quality in dense breasts [8, 16, 17]. Currently, most mammography equipment uses full field digital mammography (FFDM), which has high detection quantum efficiency. FFDM enables the acquisition of images suitable for diagnosis with the addition of image processing, even in thickened breast tissue. Such imaging has been shown to be effective in breast cancer screening in dense breasts [18].

One of the physical indicators of digital imaging quality is contrast to noise ratio (CNR) [19]. CNR is used to manage the precision of digital equipment and to compare their performance. By increasing the exposure and average glandular dose (AGD) of radiation, the MMG image quality in dense breast tissue can be improved [20]. There is, however, a trade-off relationship between image quality and exposure. To optimize image quality, especially in thick breast tissues, it is important to understand the complex relationship between the CNR and AGD in MMG. Breast-equivalent phantoms mimic the 3-dimensional structure of the human breast and offer an attractive option to study the variation of CNR and AGD with different breast thicknesses [21]. Breast phantoms are available in different thicknesses and tissue ratios corresponding to varying mammary gland densities and have been extensively used for MMG imaging studies [22, 23]. A previous study using breast phantoms showed AGD increases with increasing breast thickness [24]. Another study with breast phantoms showed that, with increased breast thickness, AGD values increase and CNR values decrease [25]. The aim of this study was to corroborate the relationship between CNR, mammary gland ratio, AGD, and phantom thickness using breast phantoms of varying thickness. We hypothesized that the correlation of AGD and CNR could be applied to clinical settings to enable the acquisition of images with an optimal trade-off between image quality and radiation dose.

The article "Effect of Different Breast Densities and Average Glandular Dose on Contrast to Noise Ratios in Full-Field Digital Mammography: Simulation and Phantom Study" was published in 2018. Journal: Radiol Res Pract.

## 2. Materials and Methods

An FFDM breast X-ray device and three types of breast-equivalent phantoms with different tissue ratios were used. The prediction formula for the CNR was calculated by multivariate analysis, and the effects of the various mammary gland densities and AGD on CNR were evaluated using a statistical analysis model.

### 2.1. Breast-Equivalent Phantoms

Breast-equivalent phantoms (Eastek Breast Phantom Research Set CI RS Model 14A, Norfolk, VA) of three mammary gland/fat tissue ratios were used: Phantom A (30/70), Phantom B (50/50), and Phantom C (70/30). By combining individual phantoms of 5-mm, 10-mm and 20-mm thicknesses, breast phantom models of seven thicknesses ranging from 10 mm to 70 mm were created. A polymethyl methacrylate phantom was arranged around the periphery of the breast model to suppress the effect of scattered radiation, and the device was configured so the detector was completely covered (Figure 1).

### 2.2. Imaging of Breast-Equivalent Phantoms

The phantoms (three tissue ratios, seven thicknesses) were imaged using FFDM (General Electric Senographe Essential F, Buc, France). Imaging was performed using the Auto Exposure Control imaging mode, which automatically selected the target/additional filter combinations (molybdenum [Mo]/Mo, Mo/rhodium [Rh], or Rh/Rh) and tube voltage for imaging. The imaging conditions (tube voltage, current time product [mAs value], and average glandular dose [AGD]) as displayed on the equipment were recorded. Each breast model was imaged thrice and the mean of each displayed value was calculated.

### 2.3. CNR Measurements and Calculation

CNR measurements were performed following the guidelines described in IEC 61223-3-2Ed.2.0 [26]. A 99.9% pure aluminum plate (CIRS T43009) measuring 100 mm × 100 mm × 0.2 mm was placed at the center of the phantom as a contrast substance. Images were acquired with and without the aluminum plate in place for each breast model. A 20 mm × 20 mm rectangular region of interest (ROI) was marked along the central line on the longitudinal axis of the X-ray for the two captured images, corresponding to the nipple side and 60 mm away from the chest wall side of the breast support table. The average pixel value within the ROI was measured in both images (with and without the aluminum plate, Figure 2) using ImageJ software (National Institutes of Health, Bethesda, MD).

CNR values were calculated from the measured pixel values according to the following previously published [27]:

(1) $$\begin{array}{c} CNR=\frac{\left(m_{BG}-m_{AL}\right)}{\sqrt{\left(\sigma_{BG}^{2}+\sigma_{AL}^{2}\right)/2}} \end{array}$$

where **m**_**AL**_ is the mean pixel value of the 20 × 20 mm ROI with the aluminum plate in position, **σ**_**AL**_^2^ is the corresponding pixel value standard deviation, **m**_**BG**_ is the mean pixel value without the aluminum plate in place, and **σ**_**BG**_^2^ is the corresponding pixel value standard deviation.

The article "Effect of Different Breast Densities and Average Glandular Dose on Contrast to Noise Ratios in Full-Field Digital Mammography: Simulation and Phantom Study" was published in 2018. Journal: Radiol Res Pract.

### 2.4. Statistical Analysis

SAS JMP ver13.1.0 (SAS Institute, Cary, NC) and Student's t test were used and p < 0.05 was considered significant for all statistical analyses. Residual sum of squares and multivariate (simple linear regression) analysis were performed with the mammary gland tissue ratio and AGD as independent variables and the CNR as the dependent variable to assess the effect of the mammary gland tissue ratio and AGD on CNR. The mean CNR at each mammary gland tissue ratio was adjusted by the AGD as a covariate and the difference in CNR values between different mammary gland tissue ratios was determined.

Next, the correlation between the AGD and the CNR was assessed for each mammary gland ratio. A strong positive correlation was defined as r ≥ 0.7. Using an Excel function, a prediction equation was obtained for each mammary gland ratio. Using the root mean square error (RMSE) analysis, prediction accuracy was assessed by comparing the predicted values of the CNR adjusted by the AGD with the actual CNR values for each mammary gland ratio.

A multivariate (least squares method) analysis was performed with the mammary gland tissue ratio (30/70, 50/50, and 70/30) and AGD as independent variables and the CNR as a dependent variable to identify the factors associated with CNR. Factors with t-values below |2.00| were defined as not contributing significantly to the CNR. Additionally, larger absolute values were defined to have a greater contribution. A predictive formula of CNR was obtained by generalizing the analysis model. Predicted and measured values of the CNR were compared using the RMSE to evaluate the accuracy of the predictive formula.

Finally, a multivariate linear regression model with the CNR as the objective variable and mammary gland ratio, AGD, and phantom thickness as the explanatory variables was constructed, with the intent to determine the correlation between the CNR and each measurement item. Additionally, analysis of variance based on the constructed multivariate linear regression model was conducted and the contribution rate for each of the variables was calculated. For the analysis of variance, the mammary gland ratio used AGD as the variable factor and phantom thickness as the continuous variable. R (v. 3.2.4) was used for this analysis (R Foundation for Statistical Computing, Vienna, Austria) and Wald Test was used to estimate the regression coefficient and 95% confidence interval.

The article "Effect of Different Breast Densities and Average Glandular Dose on Contrast to Noise Ratios in Full-Field Digital Mammography: Simulation and Phantom Study" was published in 2018. Journal: Radiol Res Pract.

## 3. Results

Table 1 and Figure 3 show the imaging conditions and CNR values calculated for the three breast models with different tissue ratios and thicknesses. CNR values were highest in Phantom A (30/70) at all thicknesses. In general, higher CNR values were obtained with lower mammary gland ratios and lower phantom thicknesses. The variation in CNR among the three breast models was low (coefficient of variation, 3.4-8.7%) at lower phantom thicknesses (10–30 mm) and increased (coefficient of variation, 10.5-16.8%) with increases in phantom thickness (50–70 mm). Notably, with a breast model thickness of 70 mm, the CNR in breast model C (70/30) was 26% lower compared to that in breast model A (30/70).

Table 2 shows the results of the multivariate analysis performed to investigate the effects of the mammary gland tissue ratio and AGD on the CNR. The p-values for the mammary gland ratio and AGD were < 0.0476 and < 0.0001, respectively, showing statistical significance. The results showed that both the mammary gland ratio and the AGD were significant predictors of CNR.

The mean CNR of each mammary gland ratio adjusted by the AGD as a covariate is shown in Table 3. The difference in CNR between mammary gland ratios is shown in Table 4. The p-value for the comparison between Phantoms A (30/70) and C (70/30) was 0.0213, showing a statistically significant difference in CNR between the two models.

Figure 4 shows that there was a strong negative correlation (r = -0.8989) between the CNR and the AGD across all three mammary gland ratios. In addition, a strong negative correlation (r = -0.8989) was also observed between the CNR and AGD at each mammary gland ratio. The prediction equations for the CNR based on the AGD values for each mammary gland ratio are provided in Table 5. The comparison between the predicted values of the CNR adjusted by AGD and the actual CNR values for each mammary gland ratio is shown in Figure 5 and Table 5. The accuracy of the CNR predicted by the mammary gland ratio was highest (r2 = 0.946, RMSE = 1.314) in Phantom B (50/50), followed by Phantom A (30/70) (r2 = 0.928, RMSE = 1.323) and Phantom C (70/30) (r2 = 0.833, RMSE = 2.301).

Based on the multivariate (least squares method) analysis of the mammary gland tissue ratio and AGD as independent variables and the CNR as a dependent variable and on generalizing the analysis model, the CNR-predictive formula was obtained as follows:

Fibroglandular adipose mass (%): 30/70

(2) $$\begin{array}{c} CNR=-10.81\times AGD+1.56+27.1 \end{array}$$

Fibroglandular adipose mass (%): 50/50

(3) $$\begin{array}{c} CNR=-10.81\times AGD-0.56+27.1 \end{array}$$

Fibroglandular adipose mass (%): 70/30

(4) $$\begin{array}{c} CNR=-10.81\times AGD-1.01+27.1 \end{array}$$

This predictive formula revealed r2 = 0.865 and RMSE = 1.893, indicating that it is possible to predict the CNR using the AGD and mammary gland ratio.

The article "Effect of Different Breast Densities and Average Glandular Dose on Contrast to Noise Ratios in Full-Field Digital Mammography: Simulation and Phantom Study" was published in 2018. Journal: Radiol Res Pract.

Table 6 shows that there was a significant correlation between the mammary gland ratio and phantom thickness and CNR (Regression coefficient 24.449, p value = 7.720E-13). The regression value was significantly lower for phantom C (Regression coefficient = -2.146, p value = 3.976E-03). The results suggest that the regression value significantly decreases as the phantom thickness increases (Regression coefficient = -0.228, p value = 8.041E-05). The phantom thickness contribution rate was 91.43%, which suggests that it can explain 91.43% of the CNR.

Table 7 shows that there was a significant correlation between the mammary gland ratio and phantom thickness and CNR (Regression coefficient = 24.629, p value = 1.038E-17). The results show that the regression value was significantly lower for phantoms B (Regression coefficient = -1.3, p value = 4.946E-02) and C (Regression coefficient = -2.157, p value = 2.684E-03). A decrease in the CNR value with an increase in phantom thickness was observed.

Table 8 shows that there was a significant correlation between the mammary gland ratio and AGD and CNR (Regression coefficient = 28.668, p value = 3.647E-13). The results suggest that the CNR value was significantly lower for phantom C (Regression coefficient = -2.559, p value = 2.178E-02). A significant decrease in the CNR value was observed along with the increase in AGD value. A comparison of the results with the Akaike's Information Criterion value, which expresses the goodness of fit of the model, showed that using phantom thickness as the explanatory variable produces a better model than using the AGD as the explanatory variable.

## 4. Discussion

In this study, we investigated the CNR and AGD of mammography using breast-equivalent phantoms with different tissue ratios and thicknesses. Our results showed that higher CNR values were obtained with breast-equivalent phantoms having lower mammary gland tissue ratios and lesser thickness. The CNR values showed a strong negative correlation with AGD values. These results corroborate previous reports of reduced cancer diagnosis sensitivity and poor MMG image quality in high-density mammary glands [13, 16, 17].

CNR is generally considered to be an index of image quality in various diagnostic imaging devices [28]. Image quality should also undergo manual evaluation, as image processing and image displays can significantly affect image quality in digital imaging equipment. Breast thickness is an important factor affecting image quality [16, 17]. The average breast thickness has been reported to vary from 37.7 mm in Japanese women [29] to 45 mm in American women, 52 mm in British women, and 56 mm in German women [30]. Most FFDM use an automatic imaging mode that automatically selects targets/additional filters based on breast thickness to optimize exposure [31]. Therefore, the effect of breast thickness on CNR is often missed. Our results can be extrapolated to such clinical situations, where the effect of breast thickness on CNR can be estimated using AGD as an explanatory variable. Our results suggest that CNR prediction based on the tissue ratio could be used as a yardstick to evaluate the diagnostic reliability of MMG in breast cancer. CNR could be used as a postprocessing index to objectively control for the effect of the mammary gland ratio and thickness on image quality and improve the reliability of diagnosis that is otherwise subjective and dependent on the mammography readers.

The article "Effect of Different Breast Densities and Average Glandular Dose on Contrast to Noise Ratios in Full-Field Digital Mammography: Simulation and Phantom Study" was published in 2018. Journal: Radiol Res Pract.

Our study findings closely relate to previous studies that show the effect of breast density on mammographic sensitivity [13, 16, 17]. These studies show that sensitivity of mammographic detection declines with increasing breast density and that adjunct screening methods like ultrasonography could be used to increase detection sensitivity. Another study that evaluated the effect of breast thickness on AGD and CNR reported results complementary to our findings [25]. They showed that with increasing breast thickness, AGD values increase and CNR values decrease. Our study extends these results and establishes a predictive formula for CNR based on AGD, which has high accuracy and precision (R2 of 0.865 and RMSE of 1.893). Our results show that both mammary gland ratio and AGD are significant predictors of CNR, with AGD having a greater effect on CNR. Interestingly, our results also show that variation of CNR within the three breast tissue models is low at low phantom thickness (10-30 mm; coefficient of variation: 3.4-8.7%) and increases with increased phantom thickness (50~70 mm; coefficient of variation: 10.5-16.8%). This suggests that breast thickness might be a strong predictor of CNR, independent of the tissue density.

Finally, multiple logistic regression analysis results showed that mammary gland ratio and phantom thickness were significantly correlated with CNR. To ensure that each variable was incorporated in the analysis model independently and to avoid inferior results from incorporating related variables into the analysis model at the same time, we conducted the regression analysis using two additional models, where the first model incorporated phantom thickness and the second model incorporated the AGD.

The article "Effect of Different Breast Densities and Average Glandular Dose on Contrast to Noise Ratios in Full-Field Digital Mammography: Simulation and Phantom Study" was published in 2018. Journal: Radiol Res Pract.

This study has several limitations. First, there is the inherent limitation of a basic research study using phantoms. Phantoms have uniform tissue ratios and do not possess the heterogeneity of mammary gland density distribution encountered in the human breast [21]. The results of this study will require clinical validation in human subjects. Second, MMG was performed using a single FFDM device; therefore, it may not be possible to directly apply or extrapolate the results to other MMG devices. Third, we used a high-contrast aluminum plate for CNR measurement and investigated only the spatial resolution aspect, but not the density resolution aspect, of contrast resolution. CNR evaluates the signal difference between the two surfaces and the noise ratio of the obtained image. Therefore, CNR is not considered to provide sharpness information. It is also essential to investigate image features like density resolution and visibility. Since ultrasound examination is known to improve diagnostic reliability in dense breasts, future studies should investigate the role of the CNR in approaches combining ultrasound examinations and MMG for breast cancer screening [32].

CNR is one of the image assessments under mammography. The CNR value cannot be obtained without using phantom. On the other hand, AGD appears on the mammography monitor under FFDM. This value can be easily obtained. Thus, applying the computation expression obtained under this research will enable us to easily obtain the CNR from the AGD value in real time immediately after mammography. Originally, the MMG observer used to make subjective evaluations based on the image contrast and noise. However, having the CNR value will enable more objective observations of images and this is anticipated to improve the diagnostic performance of cancer.

## 5. Conclusions

In this investigation we demonstrated that CNR varies inversely with mammary gland to fat tissue ratio and breast tissue thickness, which explains the clinical observation of poor MMG image quality in dense breasts. We also demonstrated a significant correlation between the CNR and the AGD based on the tissue ratio and developed a predictive formula for CNR using AGD and mammary gland density. CNR prediction based on the tissue ratio could be used as a yardstick to measure the diagnostic reliability of MMG in breast cancer, objectively control for the effect of mammary gland ratio on image quality, and improve the reliability of diagnosis that is otherwise subjective.

The article "Effect of Different Breast Densities and Average Glandular Dose on Contrast to Noise Ratios in Full-Field Digital Mammography: Simulation and Phantom Study" was published in 2018. Journal: Radiol Res Pract.

## Figures and Tables

**Figure 1:** Experimental set up of the phantom for the CNR measurement based on the International Electrotechnical Committee guidelines (a) without and (b) with the aluminum plate placed at the center of the horizontal axis of the breast support. CNR: contrast to noise ratio and PMMA: polymethyl methacrylate.

**Figure 2:** Schematic showing the region of interest (ROI) in the breast-equivalent phantom (a) without and (b) with the aluminum plate. Pixel values were calculated using ImageJ in the ROI without (BG-ROI) and with (Al-ROI) the aluminum plate.

**Figure 3:** Contrast to noise ratio (CNR) measurement results in breast phantoms with three different tissue ratios plotted against phantom thickness. The CNR was highest in phantom model A (30/70) at all thicknesses. The CNR decreased as the mammary gland density increased, and the thickness of the breast model increased. Mo: molybdenum and Rh: rhodium.

**Figure 4:** Correlation between the AGD and CNR (a) across all three mammary gland ratios, and in (b) model A (30/70), (c) model B (50/50), and (d) model C (70/30). AGD: average glandular dose and CNR: contrast to noise ratio.

**Figure 5:** Correlation between the CNR predicted value measured at different tissue ratios in (a) model A (30/70), (b) model B (50/50), and (c) model C (70/30). CNR: contrast to noise ratio. ^*∗*^Range above and below the approximate line is 95% CI.

**Table 1:** CNR values based on mammary gland density and imaging conditions.

Fibroglandular adipose mass (%)	Thickness of phantom (mm)	Target filter	Tube voltage (kV)	mAs (mAs)	AGD (mGy)	CNR
Phantom A (30/70)	10	Mo/Mo	26	16.7	0.48	23.1
	20		26	27.9	0.75	20.1
	30	Mo/Rh	27	41.7	1.01	16.2
	40		28	57.1	1.27	15.1
	50	Rh/Rh	29	60.8	1.33	13.0
	60		29	74.9	1.58	11.7
	70		30	90.2	1.95	10.9

Phantom B (50/50)	10	Mo/Mo	26	18	0.53	21.8
	20		26	34	0.85	20.8
	30	Mo/Rh	27	47.2	1.07	16.0
	40	Rh/Rh	29	50.1	1.2	13.7
	50		30	52.4	1.23	11.4
	60		31	59.7	1.49	9.6
	70		30	75	1.47	8.4

Phantom C (70/30)	10	Mo/Mo	26	19.1	0.54	21.8
	20		26	37.8	0.87	19.1
	30	Mo/Rh	27	44	0.9	13.8
	40	Rh/Rh	29	59.7	1.23	12.6
	50		30	69	1.55	10.6
	60		30	64	1.29	9.0
	70		30	95.3	1.73	8.1

AGD: average glandular dose, CNR: contrast to noise ratio, Mo: molybdenum, and Rh: rhodium.

**Table 2:** Results of the multivariate analysis for effect of mammary gland density and AGD on CNR.

Variables	Parameter	df	Sum of squares	F value	p
Mammary gland tissue ratio	2	2	26.3	3.66	0.0476
AGD	1	1	376.6	105.06	< 0.0001

AGD: average glandular dose, CNR: contrast to noise ratio, and df: Degrees of Freedom.

The article "Effect of Different Breast Densities and Average Glandular Dose on Contrast to Noise Ratios in Full-Field Digital Mammography: Simulation and Phantom Study" was published in 2018. Journal: Radiol Res Pract.

**Table 3:** Mean CNR for each mammary gland tissue ratio adjusted by the AGD as a covariate.

Breast phantom model (Fibroglandular/adipose ratio)	CNR	Unadjusted difference [95%CI]	p	CNR	Adjusted for AGD difference [95%CI]	p
A (30/70)	15.73	-1.3	0.6274	16.14	-0.92	0.1459
B (50/50)	14.43	[-6.84, 4.24]		15.22	[-2.23, 0.39]	
C (70/30)	15.73	-2.17	0.4217	16.14	-2.66	0.0017
A (30/70)	13.57	[-7.7, 3.37]		13.48	[-4.03, -1.29]	
B (50/50)	14.43	-0.87	0.7465	15.22	-1.74	0.0006
C (70/30)	13.57	[-6.4, 4.67]		13.48	[-2.5, -0.98]	

**Table 4:** Pairwise differences in the CNR between phantoms with different mammary gland ratios.

	CNR difference [95%CI]	p
A (30/70) vs. B (50/50)	-2.12 [-4.26, 0.02]	0.0521
A (30/70) vs. C (70/30)	-2.57 [-4.71, -0.43]	0.0213
B (50/50) vs. C (70/30)	-0.45 [-2.59, 1.69]	0.6637

CNR: contrast to noise ratio and CI: confidence interval.

**Table 5:** Predictive formulae for CNR according to breast density.

Breast phantom model (Fibroglandular/adipose ratio)	Correlation with CNR		CNR predictive formula	R^2^	RMSE
	r	p			
A (30/70)	-0.9631	<0.0005	CNR = -8.69×AGD+26.12	0.928	1.323
B (50/50)	-0.9724	<0.0002	CNR = -14.62×AGD+30.80	0.946	1.314
C (70/30)	-0.9126	<0.0041	CNR = -11.29×AGD+26.64	0.833	2.301

Model: p < 0.0001, R^2^ = 0.865, and RMSE = 1.893. CNR: contrast to noise ratio and RMSE: root mean square error.

**Table 6:** Results of multivariate linear regression analysis using CNR as the objective variable and mammary gland ratio, AGD, and phantom thickness as the explanatory variables.

		Regression results				Analysis of variance	
Variable	Level	Regression coefficient	Lower limit of 95% confidence interval	Upper limit of 95% confidence interval	Wald test p value	Contribution rate	Chi-squared test p value
Constant term	-	24.489	21.929	27.049	7.720E-13	-	-
Phantom type	B	-1.276	-2.665	0.112	6.911E-02	3.63%	1.213.E-02
Phantom type	C	-2.146	-3.499	-0.792	3.976E-03	-	-
Phantom thickness	-	-0.228	-0.321	-0.136	8.041E-05	91.43%	9.500.E-12
AGD	-	0.311	-4.402	5.025	8.904E-01	0.01%	8.904.E-01

AGD: average glandular dose and CNR: contrast to noise ratio.

**Table 7:** Results of multivariate linear regression analysis using CNR as the objective variable and phantom type and phantom thickness as the explanatory variables.

		Regression results				Analysis of variance	
Variable	Level	Regression coefficient	Lower limit of 95% confidence interval	Upper limit of 95% confidence interval	Wald test p value	Contribution rate	Chi-squared test p value
Constant term	-	24.629	23.228	26.029	1.038.E-17	-	-
Phantom type	B	-1.3	-2.597	-0.003	4.946.E-02	3.63%	9.247.E-03
Phantom type	C	-2.157	-3.454	-0.861	2.684.E-03	-	-
Phantom thickness	-	-0.223	-0.249	-0.196	2.108.E-12	91.43%	2.108.E-12

AIC 71.01658, CNR: contrast to noise ratio, and AIC: Akaike's Information Criterion.

The article "Effect of Different Breast Densities and Average Glandular Dose on Contrast to Noise Ratios in Full-Field Digital Mammography: Simulation and Phantom Study" was published in 2018. Journal: Radiol Res Pract.

**Table 8:** Results of multivariate linear regression analysis using CNR as the objective variable and phantom type and AGD as the explanatory variables.

		Regression results				Analysis of variance	
Variable	Level	Regression coefficient	Lower limit of 95% confidence interval	Upper limit of 95% confidence interval	Wald test p value	Contribution rate	Chi-squared test p value
Constant term	-	28.668	25.607	31.729	3.647.E-13	-	-
Phantom type	B	-2.119	-4.262	0.024	5.230.E-02	3.63%	1.305.E-01
Phantom type	C	-2.559	-4.697	-0.421	2.178.E-02	-	-
AGD	-	-10.822	-13.048	-8.595	1.070.E-08	82.96%	1.070.E-08

AIC: 99.99013, AGD: average glandular dose, and CNR: contrast to noise ratio, Akaike's Information Criterion.

## Data Availability

The imaging and other data used to support the findings of this study are included within the article.

## References

[1] Falun Meeting, Falun, Sweden O. C. (1996). Breast-cancer screening with mammography in women aged 40–49 years. *International Journal of Cancer*.

[2] Sakamoto G., Inaji H., Akiyama F. (2005). General rules for clinical and pathological recording of breast cancer 2005.. *Breast cancer (Tokyo, Japan)*.

[3] Wolfe J. N., Saftlas A. F., Salane M. (1987). Mammographic parenchymal patterns and quantitative evaluation of mammographic densities: a case-control study. *American Journal of Roentgenology*.

[4] Rice M. S., Bertrand K. A., VanderWeele T. J. (2016). Mammographic density and breast cancer risk: A mediation analysis. *Breast Cancer Research*.

[5] Mehnati P., Alizadeh H., Hoda H. (2016). Relation between mammographic parenchymal patterns and breast cancer risk: Considering BMI, compressed breast thickness and age of women in Tabriz, Iran. *Asian Pacific Journal of Cancer Prevention*.

[6] Green V. L. (2016). Mammographic breast density and breast cancer risk: Implications of the breast density legislation for health care practitioners. *Clinical Obstetrics and Gynecology*.

[7] McCormack V. A., dos Santos Silva I. (2006). Breast density and parenchymal patterns as markers of breast cancer risk: a meta-analysis. *Cancer Epidemiology Biomarkers & Prevention*.

[8] Boyd N. F., Guo H., Martin L. J. (2007). Mammographic density and the risk and detection of breast cancer. *The New England Journal of Medicine*.

[9] Yaghjyan L., Colditz G. A., Collins L. C. (2011). Mammographic breast density and subsequent risk of breast cancer in postmenopausal women according to tumor characteristics. *Journal of the National Cancer Institute*.

[10] Nagao Y., Kawaguchi Y., Sugiyama Y., Saji S., Kashiki Y. (2002). Relationship between mammographic density and the risk of breast cancer in Japanese women: A case-control study. *Breast Cancer*.

The article "Effect of Different Breast Densities and Average Glandular Dose on Contrast to Noise Ratios in Full-Field Digital Mammography: Simulation and Phantom Study" was published in 2018. Journal: Radiol Res Pract.

[11] Nagata C., Matsubara T., Fujita H. (2005). Mammographic density and the risk of breast cancer in Japanese women. *British Journal of Cancer*.

[12] Kotsuma Y., Tamaki Y., Nishimura T. (2008). Quantitative assessment of mammographic density and breast cancer risk for Japanese women. *The Breast*.

[13] Kolb T. M., Lichy J., Newhouse J. H. (2002). Comparison of the performance of screening mammography, physical examination, and breast US and evaluation of factors that influence them: an analysis of 27,825 patient evaluations. *Radiology*.

[14] D'Orsi C. J., Sickles E. A., Mendelson E. B. (2013). *ACR BI-RADS® Atlas, Breast Imaging Reporting and Data System*.

[15] Saunders R. S., Baker J. A., Delong D. M., Johnson J. P., Samei E. (2007). Does image quality matter? Impact of resolution and noise on mammographic task performance. *Medical Physics*.

[16] Destounis S., Johnston L., Highnam R., Arieno A., Morgan R., Chan A. (2017). Using volumetric breast density to quantify the potential masking risk of mammographic density. *American Journal of Roentgenology*.

[17] Kerlikowske K., Phipps A. I. (2011). Breast density influences tumor subtypes and tumor aggressiveness. *Journal of the National Cancer Institute*.

[18] Lewin J. M., Hendrick R. E., D'Orsi C. J. (2001). Comparison of full-field digital mammography with screen-film mammography for cancer detection: Results of 4,945 paired examinations. *Radiology*.

[19] Baldelli P., Phelan N., Egan G. (2009). A novel method for contrast-to-noise ratio (CNR) evaluation of digital mammography detectors. *European Radiology*.

[20] Oliveira M., Nogueira M. S., Guedes E. (2007). Average glandular dose and phantom image quality in mammography. *Nuclear Instruments and Methods in Physics Research Section A: Accelerators, Spectrometers, Detectors and Associated Equipment*.

[21] Kiarashi N., Nolte A. C., Sturgeon G. M. (2015). Development of realistic physical breast phantoms matched to virtual breast phantoms based on human subject data. *Medical Physics*.

[22] Ko M.-S., Kim H. H., Cha J. H., Shin H. J., Kim J. H., Kim M. J. (2013). Dose reduction in automatic optimization parameter of full field digital mammography: Breast phantom study. *Journal of Breast Cancer*.

[23] Kiarashi N., Lo J. Y., Lin Y. (2014). Development and application of a suite of 4-D virtual breast phantoms for optimization and evaluation of breast imaging systems. *IEEE Transactions on Medical Imaging*.

[24] Kaabi F. A., Bariki N. A., Janeczek J. Variation of the Breast Mean Glandular Doses According to Breast Thicknesses.

The article "Effect of Different Breast Densities and Average Glandular Dose on Contrast to Noise Ratios in Full-Field Digital Mammography: Simulation and Phantom Study" was published in 2018. Journal: Radiol Res Pract.

[25] Karaaslan M. K., Gundogdu O., Muzoglu N., Arici M. A. Variation of contrast-noise ratio (CNR) and mean glanduler dose according to breast thickness.

[26] Evaluation and routine testing in medical imaging departments Part 3-2: Acceptance tests - Imaging performance of mammographic X-ray equipment. International Electrotechnical Committee. 2007

[27] Matsubara K., Matsumoto C., Mochiya Y., Toda K., Noto K., Koshida K. (2014). [Radiation dose evaluation in a photon-counting digital mammography unit].. *Nihon Hoshasen Gijutsu Gakkai zasshi*.

[28] Tapiovaara M. J., Wagner R. F. (1993). SNR and noise measurements for medical imaging: I. A practical approach based on statistical decision theory. *Physics in Medicine and Biology*.

[29] Matsumoto M., Nishizawa K., Akiyama Y., Horita K., Kato H., Ishioka A. (2000). The Mean breast thickness for Japanese patients for use in estimating the glandular dose in mammography. *Journal of Japan Association of Breast Cancer Screening*.

[30] Jamal N., Ng K.-H., McLean D. (2003). A study of mean glandular dose during diagnostic mammography in Malaysia and some of the factors affecting it. *British Journal of Radiology*.

[31] Shramchenko N., Yaffe M. J., Flynn M. J., Blin P., Mathey C., Klausz R. Optimized exposure control in digital mammography.

[32] Ohuchi N., Suzuki A., Sobue T. (2016). Sensitivity and specificity of mammography and adjunctive ultrasonography to screen for breast cancer in the Japan Strategic Anti-cancer Randomized Trial (J-START): A randomised controlled trial. *The Lancet*.

